RETRACTED

# Application of the Whole Optimization of Emergency Nursing Model United and Its Influence on Patients' Stress Response and Nursing Satisfaction

**DOI:** 10.1155/2022/9936211

**Published:** 2022-05-28

**Authors:** Dannan Ai, Sumin Xu

**Affiliations:** ^1^Emergency Room, The First Affiliated Hospital of Soochow University, Suzhou, 215000 Jiangsu, China; ^2^Department of Interventional, The First Affiliated Hospital of Soochow University, Suzhou, 215000 Jiangsu, China

## Abstract

**Objective:**

To investigate the use of an integrated emergency nursing model with a multidisciplinary team (MDT) teaching method for practice of nursing towards multiple trauma in the emergency department and its influence on patients' stress response and nursing satisfaction.

**Methods:**

The research subjects were 120 multiple trauma patients hospitalized to our hospital's emergency department between January 2019 and January 2020, who were evenly divided into groups A (*n* = 60) and B (*n* = 60) based on the sequence of admission. For patients in group A, on the basis of whole optimization of the emergency nursing model, the MDT teaching and training were given to the nursing staff in group A. Patients in group B had their emergency nursing model completely optimized. The assessment scores of nursing staff were compared. The patients' C-reactive protein (CRP) levels in peripheral circulation, first-aid time indices, treatment effect, risk of complications & nursing contentment were all investigated.

**Results:**

Nursing personnel in group A had considerably higher achievement scores than staff nurses in group B (*P* < 0.001). CRP levels in group A were considerably lower following therapy (*P* < 0.05) than those in group B. The time it took for group A to receive first assistance was considerably less than that for group B (*P* < 0.001). Group A had a considerably superior treatment effect than group B (*P* < 0.05). Complications occurred at a lower rate in group A (*P* < 0.05) than in group B. Group A nurses were more satisfied than group B nurses (*P* < 0.05).

**Conclusion:**

The entire optimization of the emergency nursing model combined with the MDT way of teaching can abbreviate the rescue process, reduce stress, improve treatment effect & reduce the possibility of complications in multiple trauma patients in the emergency department, and patients seem to be more comfortable with this nursing model. As a result, it should become more well known.

## 1. Introduction

Multiple trauma patients have at least two organ injuries caused by one reason such as external force and falling accidents. In recent years, with the changes of the living environment, the number of multiple trauma patients worldwide is increasing with each passing day and patients are facing a high mortality [1–3]. Physical traumas are tragic and multifaceted injuries that suddenly threaten life. Since the multiple trauma is usually complicated, providing efficient and scientific treatment for patients is the key to protect their lives and health. In clinical practice, the patients' traumatic conditions should be made clear as soon as possible, the priority should be clarified, and the multidisciplinary team (MDT) method should be used in treatment to comprehensively improve the prognosis of patients. MDT originated in the United States in the last century, which can integrate medical resources, conduct regular meetings for specific diseases, and formulate clinical therapy plans. Patients' survival rates are enhanced with the support of interdisciplinary expertise [4–7]. At present, MDT is often used in neurosurgical diseases and respiratory diseases but rarely used in the research of multiple trauma treatment in academic circles. However, clinical practice shows that the general emergency nursing process for multiple trauma patients is very complicated and the subjective initiative of nursing staff is poor. So, the treatment effect of patients still needs to be further improved [8–11]. As a result, the purpose of this article is to investigate the use of the whole optimization of the emergency nursing model in conjunction with the MDT teaching technique in the nursing practice of multitrauma in the emergency unit and its influence on patients' stress response and nursing satisfaction. The research subjects were 120 multiple trauma sufferers hospitalized to our hospital's emergency department between January 2019 and January 2020, with the following summary.

RETRACTED

## 2. Materials & Methods

### 2.1. General Data

The research subjects were 120 multiple trauma patients who were hospitalized to our hospital's emergency unit between January 2019 & January 2020 that were evenly divided into groups A (*n* = 60) & B (*n* = 60) based on the sequence of admission. There was no substantial difference in general information among the two groups (*P* > 0.05). The hospital's ethics committee authorized this study.

### 2.2. Inclusion Criteria

The following were the study's inclusion criteria: (1) the participants or their relatives were fully told about the study & completed the written informed consent; (2) after assessment, the patients satisfied the criteria for multiple trauma [12]; (3) the trauma severity scores of the patients were higher than 16 [13]; and (4) the patients were seen within 12 hours after the accident.

### 2.3. Exclusion Criteria

The exclusion criteria of patients in this study were as follows: (1) the patients with mental problems or who were unable to communicate with others; (2) the patients who were suffering from other diseases; (3) the sufferers who received treatment in other hospitals before coming to our hospital; and (4) the patients who had contraindications to surgery [14].

### 2.4. Methods

For patients in group A, on the basis of whole optimization of the emergency nursing model, the MDT teaching and training were given to the nursing staff among group A. The following were the precise steps: (1) The MDT emergency rescue nursing teams were set up, with 3 nurses in each team. The situational questions were designed according to the actual treatment of emergency multiple trauma and included the following: (a) the patients' symptoms and severity of the disease, including risk factors, potential risks, emergency care plans, complications, and key observation directions, and (b) basic nursing measures and rescue process of patients. (2) According to the situational questions, nursing staff should consult relevant literature and adopt the evidence-based nursing model to put forward solutions to them. (3) Nursing staff should communicate with each other within the team, master the nursing methods for multiple trauma patients in the emergency department, learn each other's strong points, make up for their weak points in the process of communication, and play a role of mutual inspiration. Teachers should guide and help the nursing staff to combine evidence-based information with the situation of the emergency department, so as to deepen the nursing staff's impression on the knowledge that they have learned. (4) After teaching, the nursing staff should apply the knowledge that they have learned to practice. Each team member held one position, namely, trauma care staff, circulation nursing staff, and coordinating nursing staff. Among them, trauma care staff were the senior nurses and mainly responsible for the teams' collaboration. Circulation nursing staff were mainly responsible for infusion, blood drawing, urethral catheterization, and other routine nursing measures and closely monitored the patients' physical signs. Coordinating nursing staff should clearly understand the patients' trauma classification, send samples for examination, and make preparations for the placement of first aid supplies. (5) The multiple-trauma patients should be rescued immediately after admission. The coordinating nursing staff should ask about the causes of the injuries, start the MDT nursing process, and ensure all nursing staff were in place. The nursing team should carefully assess the patients' trauma and inform the results to doctors. We carry out rescue nursing under the guidance of doctors to ensure the patients' smooth breathing. If the patients had bleeding, shock, etc., the nursing staff should immediately give them hemostasis and fluid infusion, so as to help them to control the wound and maintain systemic circulation. (6) The MDT team can assist in surgery and send patients to the trauma center for treatment after surgery.

RETRACTED

Patients in group B received whole optimization of the emergency nursing model, with specific steps as follows. (1) The prehospital emergency staff should call the nursing staff of the emergency department for patients' detailed information to make them well prepared for treatment. Emergency department nursing staff should immediately evaluate the patients' condition after admission and send the patients with severe trauma to the emergency room, with implementation of “first treatment and then payment.” (2) If the multiple-trauma patients were in a critical condition, the emergency department should set up a team with 3 nurses. The senior nurse provided guidance to manage patients' respiratory and circulatory systems and closely monitor the changes of physical signs, while the junior nurse dealt with the patients' external wounds to strengthen the collaboration ability.

### 2.5. Observation Criteria

1. The assessment scores. It included the basic theory score, emergency treatment score (case analysis, use of first aid equipment, nursing operation, and team cooperation), and comprehensive ability score. The comprehensive ability score means that patients have the ability to live dependently. A higher score represented better performance
2. The CRP levels. The patients' CRP levels were compared before and after nursing
3. The first aid time indexes. It included residence time in the emergency room, examination time, and arrival time of nursing staff and doctors in the emergency department [15]
4. The treatment effect. If the patients' indexes returned to normal, it was recovered. If the patients' indexes basically returned to normal and the physiological function was obviously enhanced, it was improved. If the patients' physical signs were not improved, it was invalid. The patients' cure rate was calculated (number of cured patients = recovered patients plus improved patients) [16]
5. The probability of complications. Hypovolemic shock, acute renal failure, acute respiratory distress syndrome & wound infection were among the problems, as well as the proportion of persons who had complications was statistically significantly noted [17]
6. Nursing satisfaction. The self-designed scale in our hospital was used for grading. If the patients gave 5 stars, it was very satisfied. If the patients gave 3–4 stars, it was satisfied. If the patients gave 2 or less stars, it was unsatisfied. The number of patients who were satisfied with nursing was statistically recorded

RETRACTED

### 2.6. Statistical Processing

The data processing program used in this work was SPSS20.0, and the drawing program was GraphPad Prism 7 (GraphPad Software, San Diego, USA). The *χ*^2^ test & the *t*-test were used to analyze count & measurement data in this investigation. The difference was significant when *P* = 0.05 was used.

## 3. Results

### 3.1. Comparison of the Assessment Scores of Nursing Staff

As indicated in Table 1, the assessment ratings of staff nurses in group A were substantially higher than in group B (*P* < 0.001).

### 3.2. The CRP Contents of Subjects Are Compared

As demonstrated in Figure 1, the CRP level of individuals in group A was considerably lower than that of individuals in group B after therapy (*P* < 0.05).

Note that the horizontal axis in Figure 1 represented before & after intervention, while the vertical axis indicated the CRP level (mg/L) spanning left to right. Group A was symbolized by the line with dots, whereas group B was represented by the line with rectangles.

Before treatment, the CRP level was 20.98 ± 3.68 mg/L in group A and 21.11 ± 3.54 mg/L in group B, with comparison among 2 groups (*t* = 0.197, *P* = 0.844). After treatment, the CRP level was 14.21 ± 3.15 mg/L in group A and 16.98 ± 5.32 mg/L in group B, with comparison among 2 groups (*t* = 3.470, *P* = 0.001). ∗ indicated that *P* < 0.05.

### 3.3. Comparison of the First Aid Time Indexes of Patients

As demonstrated in Table 2, the first aid time of individuals in group A was considerably shorter than that of patients in group B (*P* < 0.001).

### 3.4. Patients' Treatment Effects Are Compared

As demonstrated in Table 3, the therapeutic effectiveness of individuals in group A was substantially better than that of individuals in group B (*P* < 0.05).

### 3.5. Patients' Incidence of Complications Is Compared

As demonstrated in Figure 2, the frequency of sequelae among individuals in group A was considerably lower than that of group B (*P* < 0.05).

With a comparison of the two groups (*χ*^2^ = 18.639, *P* ≤ 0.001), there were 8 instances of hypovolemia in group A and 30 cases in group B. There were 2 cases of acute respiratory distress syndrome in group A & 8 cases in group B, in comparison among the two groups (*χ*^2^ = 3.927, *P* = 0.048). There was 1 case of acute renal failure in group A & 7 cases in group B, with comparison among the two groups (*χ*^2^ = 4.821, *P* = 0.028). There were 4 cases of wound infection in group A & 12 cases in group B, with comparison flanked by the two group (*χ*^2^ = 4.615, *P* = 0.032).

RETRACTED

### 3.6. Comparison of Patients' Nursing Satisfaction

As demonstrated in Figure 3, the nurse contentment of individuals in group A was substantially greater than that of individuals in group B (*P* < 0.05).

Note that the horizontal line in Figure 3 represented extremely satisfied, satisfied, and not satisfied, while the vertical axis indicated the number of patients, from left to right (cases). Group A was represented by the black region, whereas group B was represented by the grey area. Nursing satisfaction was high in 32 cases in group A & 18 cases in group B. Nursing fulfilled 26 instances in group A & 32 cases in group B. With a comparison of the two groups (*χ*^2^ = 5.926, *P* = 0.015), two cases in group A & 10 cases in group B were not happy with nursing. The asterisk (^∗^) denotes a significance level of 0.05.

## 4. Discussion

In recent years, with the changes in people's living environment, multiple trauma caused by public security incidents or traffic accidents has become more and more common. This disease is critical and severe, which can cause circulatory disorders and immune dysfunction. In severe cases, patients may have multiple organ failure and face a high risk of death [18–21]. At present, the emergency first aid mode in practice is relatively single and lacks pertinence. Patients still need to wait for a long time after being admitted to the emergency department. The waiting time of some patients is even more than 1 hour, which seriously delays the optimal surgical time and increases mortality of patients. With the deepening of people's cognition of emergency nursing, advanced nursing models such as green channels and one-stop rescue have been applied in clinical practice. Practical results show that high-quality emergency nursing can greatly shorten the waiting time of patients, simplify the rescue process, and enable patients to receive the most efficient and scientific nursing in a short time.

In addition, this paper made an intensive study on the MDT teaching method. MDT refers to multidisciplinary cooperation for treatment, which is based on evidence-based nursing, is aimed at combining practice with theory, and deduces the most suitable nursing model for a specific disease [22–24]. The MDT teaching method can enhance the mastery of emergency nursing for multiple trauma and improve the core literacy of nursing staff. Thus, the assessment scores of nursing staff were substantially greater in group A than in group B (*P* < 0.001). The nursing team in group care is guided by evidence-based nursing-adopted cooperation based on division of labor to formulate a more efficient and scientific emergency nursing plan for multiple trauma. As a result, the time it took for individuals in group A to be rescued was shorter. Patients got timely treatment in the optimal operation time, and the overall treatment effect was better.

RETRACTED

The CRP value of individuals in group A was considerably lower after therapy than that of individuals in group B (*P* < 0.05), according to this study. CRP is an acute-phase protein. When patients are seriously injured, the secretion rate of CRP will continue to rise. Multiple-trauma victims had much higher CRP levels than healthy persons, and the more serious the body tissue damage is, the higher the CRP level is. Therefore, the decrease of the CRP level means that the stress response is alleviated, indicating that this kind of high-quality nursing model can weaken the stress response due to pain and is conducive to the recovery of patients.

Patients in group A had a considerably reduced rate of complications than those in group B (*P* < 0.05), because patients in group A received more careful nursing. The evidence-based questions raised by MDT include risk factors and potential risks for multiple-trauma patients. Through literature review combined with practical experience, nursing staff can summarize the common complications, summarize the corresponding treatment plans, and improve their ability to identify risk factors, thereby reducing the possibility of complications in patients. In the study of scholar Borns et al., multiple-trauma patients of the experimental group received high-quality nursing of the multidisciplinary team. The control group, on the other hand, got conventional emergency nursing care. The results revealed that the experimental group had a 25.0 percent (25/100) incidence of complications, which was considerably lower than the control group (*P* < 0.05) [25], demonstrating that this emergency treatment model had a positive preventative impact.

Nursing satisfaction was substantially greater in group A than in group B due to improved recuperation & reduced waiting times. It demonstrates that high-quality crisis nursing could not only enhance patient outcomes but also lower the likelihood of nurse-patient conflicts, which is beneficial to the midwife interaction [26]. However, there are also limits of this study. First, the number of patients is not large enough. Second, the mechanism of this study is not clarified, which needs further study.

## 5. Conclusion

In summary, the whole optimization of the emergency nursing model combined with the MDT teaching method can shorten the rescue process, reduce the stress response, improve the treatment effect, and reduce the possibility of complications of multiple-trauma patients in the emergency department and patients are more satisfied with this kind of nursing model [27]. Therefore, it should be popularized in practice.

RETRACTED

## Figures and Tables

**Figure 1:** CRP levels of participants were compared (−*x* ± *s*, mg/L).

**Figure 2:** Incidence of patient problems in comparison. Image 2 black region represented hypovolemic shock, the dark-gray region represented acute respiratory distress syndrome, the light-gray area represented acute renal failure, and the white area represented wound infection. (a) Group A; (b) group B.

**Figure 3:** Comparison of nursing satisfaction in patients.

**Table 1:** Nursing staff assessment ratings are compared (−*x* ± *s*, points).

Items	*n*	Basic theory	Emergency treatment	Comprehensive ability
Group A	60	80.21 ± 3.56	83.65 ± 5.21	85.12 ± 3.26
Group B	60	76.11 ± 3.57	75.26 ± 5.32	76.68 ± 3.56
*t*		6.299	8.728	13.543
*P*		0.014	0.002	0.001

**Table 2:** Comparison of first aid time indexes of patients (−*x* ± *s*, min).

Items	*n*	Residence time in emergency room	Examination time	Arrival time of nursing staff	Arrival time of doctors
Group A	60	37.59 ± 8.45	20.95 ± 3.65	6.18 ± 2.65	15.98 ± 3.65
Group B	60	56.94 ± 12.51	42.11 ± 7.26	9.68 ± 3.15	22.59 ± 5.78
*t*		9.928	20.171	6.586	7.490
*P*		0.001	0.000	0.013	0.006

**Table 3:** Comparison of treatment effect of patients (*n* (%)).

Items	*n*	Recovered	Improved	Invalid	Cure rate
Group A	60	48 (60.0)	6 (10.0)	6 (10.0)	54 (90.0)
Group B	60	36 (60.0)	6 (10.0)	18 (30.0)	42 (70.0)
*χ* ^2^		5.714	0.000	7.500	7.500
*P*		0.017	1.000	0.006	0.006

## Data Availability

The corresponding author may provide the information used to substantiate this work upon demand.
